# LncRNA MEG3 Protects Chondrocytes From IL-1β-Induced Inflammation *via* Regulating miR-9-5p/KLF4 Axis

**DOI:** 10.3389/fphys.2021.617654

**Published:** 2021-03-11

**Authors:** Yijiang Huang, Daosen Chen, Zijian Yan, Jingdi Zhan, Xinghe Xue, Xiaoyun Pan, Huachen Yu

**Affiliations:** ^1^Department of Orthopaedics, The Second Affiliated Hospital and Yuying Children’s Hospital of Wenzhou Medical University, Wenzhou, China; ^2^Key Laboratory of Orthopaedics of Zhejiang Province, Wenzhou, China

**Keywords:** inflammation, apoptosis, proliferation, OA, KLF4, miR-9-5p, MEG3

## Abstract

**Background:**

Osteoarthritis (OA) is a chronic degenerative disease of the joints characterized by articular cartilage damage, subchondral bone remodeling, osteophyte formation, and inflammatory changes. This work aims to investigate the protective role of long non-coding RNA (lncRNA) maternally expressed 3 (MEG3) against the apoptosis of chondrocytes.

**Methods:**

Chondrocyte cell lines, CHON-001, and ATDC5 were treated with different doses of interleukin-1β (IL-1β) to mimic the inflammatory response during OA pathogenesis. Quantitative real-time polymerase chain reaction was performed to measure MEG3, miR-9-5p, and Krüppel-like factor 4 (KLF4) mRNA expression levels. MEG3 and KLF4 overexpression plasmids, MEG3 shRNA, miR-9-5p mimics, and miR-9-5p inhibitors were transfected into the cells. Cell counting kit-8, wound healing assay, and flow cytometry were conducted to determine cell viability, migration, and apoptotic rate. Dual-luciferase reporter assay was adopted to verify the targeting relationships among MEG3, miR-9-5p, and KLF4. Western blot was used to detect KLF4 protein expression. Enzyme-linked immunosorbent assay was employed to measure the levels of inflammatory factors.

**Results:**

MEG3 expression in chondrocytes was down-regulated by the stimulation of IL-1β, and MEG3 negatively regulated miR-9-5p expression but positively regulated KLF4 expression. MEG3 overexpression strengthened the viability and migration of CHON-001 and ATDC5 cells but restrained the apoptosis and inflammatory response, while MEG3 knockdown had opposite effects. miR-9-5p inhibition or KLF4 overexpression could counteract the effects of MEG3 knockdown on chondrocytes. Besides that, MEG3 was proved to be a molecular sponge for miR-9-5p, and KLF4 was verified as the target of miR-9-5p.

**Conclusion:**

MEG3 can promote chondrocyte proliferation and migration and inhibit apoptosis and inflammation by sponging miR-9-5p to induce KLF4 expression, which provides a promising therapy target for OA treatment.

## Introduction

Osteoarthritis (OA) is the most common chronic joint disease featured with articular cartilage degeneration, inflammatory reaction, and osteophyte formation (Loeser et al., 2012). It is reported that OA is with high morbidity in the elderly over 65 years old, and its incidence is on the rise with the aging of the global population (Loeser et al., 2012; Sherwood, 2019). Interleukin-1β (IL-1β) is an important inflammatory factor and can play a role in the initiation and early progression of OA (Daheshia and Yao, 2008). Reportedly, chondrocytes exposed to IL-1β will release inflammatory factors and mediators, such as interleukin-6 (IL-6), interleukin-8 (IL-8), and tumor necrosis factor-α (TNF-α), which will aggravate the pathogenesis of OA (Kapoor et al., 2011).

Long non-coding RNAs (lncRNAs) are non-coding RNAs exceeding 200 nt. Many lncRNAs are implicated in regulating cartilage function and OA progression, such as SNHG1, OIP5-AS1, and maternally expressed 3 (MEG3) (Lei et al., 2019; Wang A. et al., 2019; Zhi et al., 2020). Besides that, MEG3 is considered as an important regulatory factor in many tumors, such as melanoma, pituitary tumor, and osteosarcoma (He et al., 2017). MEG3 expression is reported to be dysregulated during OA development (Wang A. et al., 2019). However, the function and regulatory mechanism of MEG3 in OA have not been fully explored.

Notably, lncRNAs can act as competitive endogenous RNAs (ceRNAs) that competitively bind to target microRNAs (miRNAs, miRs) to indirectly regulate mRNAs’ expression (Tay et al., 2014), thus participating in the occurrence and development of OA (Wang A. et al., 2019). miRNAs are a class of small non-coding RNAs, abnormally expressed in OA, and are pivotal regulators in the proliferation, apoptosis, osteogenic differentiation, and inflammatory response of chondrocytes during OA pathogenesis (Swingler et al., 2012). It is reported that miR-9-5p can inhibit chondrocyte apoptosis and promote cartilage remodeling in OA (Chen et al., 2019a). The underlying regulatory between MEG3 and miR-9-5p warrants further investigation.

Krüppel-like factor 4 (KLF4) is an important transcription factor, which can regulate the stemness of cells and other biological processes, and its dysfunction partakes in the pathogenesis of many diseases (Tanaka et al., 2014; Ghaleb and Yang, 2017). Specifically, it is reported that KLF4 expression is down-regulated in the cartilage of the patients with OA (Fisch et al., 2018). Furthermore, KLF4 expression is markedly decreased in ATDC5 cell line treated with lipopolysaccharide (Fan et al., 2019).

In the present study, chondrocytes treated with IL-1β were used to construct an *in vitro* model of OA. We explored the role of MEG3 in IL-1β-induced injury of chondrocytes and its potential mechanisms. We demonstrated that MEG3 and KLF4 expression levels were remarkably down-regulated in chondrocytes stimulated with IL-1β, while miR-9-5p expression level was increased. MEG3 could promote cell proliferation and migration but inhibit cell apoptosis and inflammation. Moreover, MEG3 could directly bind to miR-9-5p and positively regulate KLF4 expression. Our findings substantiated the function of the MEG3/miR-9-5p/KLF4 axis in OA and helped clarify the mechanism of OA progression.

## Materials and Methods

### Cell Culture and Treatment

CHON-001, ATDC5, and HEK293 cells were purchased from the American Type Culture Collection (Manassas, VA, United States) or China Center for Type Culture Collection (Wuhan, China) and cultured in Dulbecco’s modified Eagle’s medium (12430104, Gibco, Grand Island, NY, United States) with 10% fetal bovine serum (12483020, Gibco, Grand Island, NY, United States), 100 U/ml penicillin, and 100 μg/ml streptomycin (15140122, Gibco, Grand Island, NY, United States) in 5% CO_2_ at 37°C. CHON-001 and ATDC5 cell lines were stimulated with recombinant human IL-1β (SRP6169, Sigma-Aldrich, St. Louis, MO, United States) at concentrations of 1, 5, and 10 ng/ml, respectively, for 12 h to establish an *in vitro* model of OA.

### Cell Transfection

The MEG3 overexpression plasmid (pcDNA3.1–MEG3), MEG3 small interfering RNA (siRNA), KLF4 overexpression plasmid (pcDNA3.1–KLF4), miR-9-5p mimics, and miR-9-5p inhibitors and their negative controls (miR-NC) were obtained from RiboBio (Guangzhou, China). Cell transfection was performed with Lipofectamine 3000 (L3000001, Invitrogen, Carlsbad, CA, United States) according to the manufacturer’s protocol.

### Quantitative Real-Time Polymerase Chain Reaction

Total RNA was isolated from cells by TRIzol reagent (15596018, Invitrogen, Carlsbad, CA, United States). In line with the manufacturer’s protocol, 1 μg of RNA was reversely transcribed into cDNA using the first-strand cDNA synthesis kit (K1651, Invitrogen, Carlsbad, CA, United States). Quantitative real-time polymerase chain reaction (qRT-PCR) was performed on SmartChip^TM^ Real-Time PCR System (640022, TaKaRa, Dalian, China) with SYBR^®^ Premix Ex TaqTM II (DRR041A, TaKaRa, Dalian, China). The relative quantification was performed with 2^−ΔΔCt^ method using U6 and GAPDH as endogenous references. The primer sequences are listed in Table 1.

**TABLE 1:** The primers used in this study.

	**Forward**	**Reverse**
MEG3	5′-CTGCCCCATCTACACTACG-3′	5 ′-CTCCTCCGCGTCTGC TAGGGCT-3 ′
MiR-9-5p	5′-GGAGTCCGTGTGTCTGTGTG-3′	5′-GCTTTATGACGGCTCT GTGG-3′
KLF4	5′-CGGGCTGATGGGCAAGTT-3′	5′-GGGCAGGAAGGATGG GTAA-3′
GAPDH	5′-TGCACCACCAACTGCTTAGC-3′	5′-GGCATGCACTGTGGTC ATGAG-3′
U6	5′-GCTTCGGCAGCACATATACT AAAAT-3′	5′-CGCTTCACGAATTTGC GTGTCAT-3′

### Cell Viability Assay

Cell counting kit-8 assay (CCK-8, C0038, Beyotime, Shanghai, China) was employed to analyze cell viability. To be specific, cells were transferred into a 96-well plate (2,000 cells/well). After IL-1β treatment, chondrocytes were cultured for 72 h. Then, the cells were incubated with 10 μl of CCK-8 reagent at 37°C for another 2 h. After that, the OD_450nm_ of the cells was measured by a microplate reader (Bio-Rad Laboratories, Hercules, CA, United States). Cell viability (%) = absorbance (treated well)/absorbance (control well) × 100%.

### Flow Cytometry

When the cell confluence reached about 80%, the cells were treated with IL-1β for 72 h. Then, the cell apoptosis rate of the chondrocytes was measured by Annexin V-FITC/propidium iodide (PI) Apoptosis Detection Kit (C1062S and ST512, Beyotime, Shanghai, China). In brief, CHON-001 and ATDC5 cells were washed, resuspended with the binding buffer, and stained with Annexin V-FITC staining solution and PI staining solution for 30 min at room temperature in the dark. Subsequently, a flow cytometer (FacsCalibur; Becton Dickinson, Franklin Lakes, NJ, United States) was used to analyze the apoptosis rate.

### Western Blot

The total proteins of the cells were isolated by a radioimmunoprecipitation assay buffer (P0013E, Beyotime, Shanghai, China) and then quantified by a bicinchoninic acid protein assay kit (P0012, Beyotime, Shanghai, China). After the loading buffer was added, the proteins were denatured in boiling water. The protein samples were separated by 10% sodium dodecyl sulfate-polyacrylamide gel electrophoresis and then transferred onto a polyvinyl fluoride membrane (Millipore, Bedford, MA, United States). After that, the membrane was blocked in 5% skim milk for 30 min at room temperature. Next, the proteins were incubated with primary antibodies anti-KLF4 (ab214666, Abcam, Cambridge, United Kingdom) and anti-GAPDH (ab8245, Abcam, Cambridge, United Kingdom) overnight at 4°C and then incubated with the secondary antibody (ab6789, Abcam, Cambridge, United Kingdom) at room temperature for 1 h. Lastly, the protein bands were visualized using ECL chemiluminescence solution (P0018FS, Beyotime, Shanghai, China), and then, the gray value of the bands was quantified by Image Lab^TM^ Software.

### Wound Healing Assay

The transfected cells were inoculated into a six-well plate. When the bottom of the wells was covered with the cells, a cell-free area was created by scraping the cell layer with a 200-μl pipette (the pipette tip is held completely perpendicular to the plate). Then, the cells were cultured in serum-free medium for 24 h, and wound closure at 0 and 24 h was measured under a microscope and analyzed with Image Pro Plus software.

### Enzyme-Linked Immunosorbent Assay

The concentrations of IL-6, IL-8, and TNF-α in the cell culture supernatant of each group were detected by a corresponding enzyme-linked immunosorbent assay (ELISA) kit (SEKH-0013-96T, SEKH-0016-96T, and SEKH-0047-48T, Solarbio, Beijing, China). After the cell supernatant was collected, horseradish peroxidase-labeled detection antibody was added to each well (including standard wells and sample wells), and the absorbance of each well at a wavelength of 450 nm was measured. The actual concentration of the sample was calculated based on the linear regression curve of the standard sample.

### Luciferase Reporter Assay

The wild type (WT) and mutant of the MEG3 and KLF4 sequence containing the miR-9-5p binding site was designed by Sangon Biotech (Shanghai, China) and cloned into pGL3−Basic luciferase reporter vector (E1751, Promega, Madison, WI, United States) to construct the reporter vectors. MiR-9-5p mimics or control miRNAs were co-transfected into HEK293 cells with the above-mentioned reporter vectors by Lipofectamine 3000 (L3000001, Invitrogen, Carlsbad, CA, United States), respectively. At 48 h later, the relative luciferase activity of the cells in each group was analyzed by adopting the Dual-Luciferase Reporter Assay System (E1910, Promega, Madison, WI, United States).

### Statistical Analysis

All experiments were repeated at least three times. SPSS 18.0 (SPSS Inc., Chicago, IL, United States) was adopted for statistical analysis, and all data were expressed as mean ± standard deviation. Student’s *t*-test or one-way ANOVA (with Turkey’s *post hoc* analysis) was used for the comparison between/among groups. *P* < 0.05 was statistically meaningful.

## Results

### IL-1β-Induced Inflammatory Injury of Chondrocytes *in vitro*

To establish the OA model *in vitro*, diverse concentrations of IL-1β (1, 5, and 10 ng/ml) were used to treat chondrocyte cell lines CHON-001 and ATDC5 to induce inflammatory injury. The CCK-8 assay unmasked that the 5- and 10-ng/ml IL-1β treatments significantly decreased the cell viability of the chondrocytes (Figures 1A,B). Additionally, the IL-1β treatment increased the apoptosis rate of the chondrocytes and elevated the contents of IL-6, IL-8, and TNF-α in both cell lines (Figures 1C–F). In the follow-up experiments, IL-1β at 10 ng/ml was selected to stimulate chondrocytes to construct an OA model *in vitro.*

**FIGURE 1:** IL-1β-induced inflammatory injury of chondrocytes *in vitro*. **(A,B)** The viability of CHON-001 and ATDC5 cells was decreased in the 5- and 10-ng/ml IL-1β group. **(C)** The apoptosis rate of CHON-001 and ATDC5 cells was increased in the 5- and 10-ng/ml IL-1β group. **(D–F)** The levels of IL-6, IL-8, and TNF-α in CHON-001 and ATDC5 cells were increased in the 5- and 10-ng/ml IL-1β treatment group. Compared with the control, **P < 0.01 and ***P < 0.001.

### Overexpressed MEG3 Could Promote Viability and Migration but Inhibit the Apoptosis and Inflammation of Chondrocytes

The qRT-PCR implied that MEG3 expression was significantly down-regulated in CHON-001 and ATDC5 cell lines treated with IL-1β (Figure 2A). In comparison to the group transfected with pcDNA3.1–NC, MEG3 expression was markedly raised in chondrocytes transfected with pcDNA3.1–MEG3 (Figure 2B). The CCK-8 assay and wound healing assay manifested that the viability and migration ability of chondrocytes in the MEG3 overexpression group were observably higher than those in the control group (Figures 2C–E). Flow cytometry analysis and ELISA indicated that the apoptosis rate and IL-6, IL-8, and TNF-α levels in the pcDNA3.1–MEG3 group were markedly lower than those in the pcDNA3.1–NC group (Figures 2F–I). These data indicated that MEG3 expression was downregulated in the OA model *in vitro* and that overexpressed MEG3 could promote the viability and migration and restrain the apoptosis and inflammation of chondrocytes.

**FIGURE 2:** Overexpressed MEG3 could promote viability and migration but inhibit apoptosis and inflammation of chondrocytes. **(A)** The expression of MEG3 was downregulated in CHON-001 and ATDC5 cells treated with IL-1β (10 ng/ml). **(B)** The expression of MEG3 was upregulated in MEG3 overexpression models. **(C,D)** Overexpression of MEG3 could promote cell proliferation, which was validated by CCK-8 assay. **(E)** Overexpression of MEG3 could promote cell migration, which was validated by Transwell assay. **(F)** Overexpression of MEG3 could inhibit cell apoptosis, which was examined by flow cytometry. **(G–I)** Overexpression of MEG3 could decrease the levels of IL-8, IL-6, and TNF-α in chondrocytes. Compared with the control group or pcDNA3.1–NC, **P < 0.01 and ***P < 0.001.

### MEG3 Knockdown Could Inhibit Viability and Migration but Promote Apoptosis and Inflammation of Chondrocytes

The expression of MEG3, compared with that in the si-NC group, was significantly decreased in chondrocytes transfected with si-MEG3 (Figure 3A). The CCK-8 assay and wound healing assay elucidated that the viability and migration of chondrocytes with MEG3 knockdown were markedly inhibited (Figures 3B–D). The apoptosis rate and IL-6, IL-8, and TNF-α levels in the si-MEG3 group were demonstrably higher than those in the si-NC group (Figures 3E–H). These data indicated that MEG3 knockdown could inhibit viability and migration but promote apoptosis and inflammation of chondrocytes. These demonstrations further validated that MEG3 was a crucial regulator in the injury of chondrocytes.

**FIGURE 3:** MEG3 knockdown could inhibit viability and migration but promote apoptosis and inflammation of chondrocytes. **(A)** The expression of MEG3 was downregulated in MEG3 knockdown models. **(B,C)** MEG3 knockdown could inhibit cell proliferation, which was validated by CCK-8 assay. **(D)** MEG3 knockdown could inhibit cell migration, which was validated by Transwell assay. **(E)** MEG3 knockdown could promote cell apoptosis, which was examined by flow cytometry. **(F–H)** MEG3 knockdown could increase the levels of IL-6, IL-8, and TNF-α. Compared with si-NC, *P < 0.05 and **P < 0.01.

### MEG3 Repressed miR-9-5p Expression in Chondrocytes

Subsequently, LncBase Predicted v2 database was searched, and it was found that MEG3 contained a binding sequence for miR-9-5p (Figure 4A). The luciferase reporter assay depicted that the co-transfection of miR-9-5p mimics could remarkably reduce the luciferase activity of MEG3-WT reporter, but it had no evident effects on that of MEG3-MUT reporter (Figure 4B). The qRT-PCR manifested that miR-9-5p expression was remarkably raised in chondrocytes stimulated by IL-1β (Figure 4C). Additionally, the up-regulation of MEG3 expression could down-regulate miR-9-5p expression in chondrocytes, while MEG3 knockdown had the opposite effect (Figures 4D,E). These data suggested that MEG3 could target miR-9-5p and repress its expression in chondrocytes.

**FIGURE 4:** MEG3 negatively regulated miR-9-5p expression. **(A)** Bioinformatics was used to predict the binding site between miR-9-5p and MEG3. **(B)** Luciferase reporter assay verified that MEG3 could bind to miR-9-5p. **(C)** MiR-9-5p was downregulated in chondrocytes stimulated by IL-1β. **(D)** Overexpression of MEG3 could decrease miR-9-5p expression. **(E)** MEG3 knockdown could increase miR-9-5p expression. Compared with miR-NC, control, pcDNA3.1–NC, or si-NC, **P < 0.01 and ***P < 0.001.

### MiR-9-5p Could Reverse the Impact of MEG3 on Viability, Migration, Apoptosis, and Inflammation of Chondrocytes

To further clarify the function of the MEG3/miR-9-5p axis in OA, rescue experiments were performed. As against miR-NC, the qRT-PCR showed that miR-9-5p expression was observably reduced after ATDC5 and CHON-001 cells were transfected with miR-9-5p inhibitor (Figure 5A). Subsequently, the CCK-8 assay, wound healing assay, flow cytometry analysis, and ELISA assays were performed, the results of which indicated that the inhibitory effects of MEG3 knockdown on cell viability and cell migration and the promoting effect on apoptosis and inflammation were partly counteracted by miR-9-5p inhibitor (Figures 5B–H). These results revealed that the function of MEG3 on chondrocytes was mediated by its regulatory function on miR-9-5p.

**FIGURE 5:** MiR-9-5p could reverse the effects of MEG3 on chondrocytes. **(A)** MiR-9-5p expression was successfully inhibited in chondrocytes transfected with miR-9-5p inhibitor. **(B,C)** MiR-9-5p inhibitor could reverse the effects of MEG3 knockdown on the viability of chondrocytes. **(D)** MiR-9-5p inhibitor could reverse the effects of MEG3 knockdown on the migration of chondrocytes. **(E)** MiR-9-5p inhibitor could reverse the effect of MEG3 knockdown on the apoptosis of chondrocytes. **(F–H)** MiR-9-5p inhibitor could reverse the effects of MEG3 knockdown on the release of IL-6, IL-8, and TNF-α of chondrocytes. Compared with miR-NC, si-NC, or si-MEG3, *P < 0.05, **P < 0.01, and ***P < 0.001.

### KLF4 Was the Target of miR-9-5p and Its Expression Could Be Positively Modulated by MEG3

Bioinformatics analysis predicted that KLF4 was a candidate target of miR-9-5p. The luciferase reporter assay confirmed that miR-9-5p could remarkably diminish the luciferase activity of KLF4-WT reporter but had no effect on that of KLF4-MUT reporter (Figure 6A). Furthermore, KLF4 mRNA and protein expressions were markedly decreased in CHON-001 and ATDC5 cell lines stimulated by IL-1β (Figure 6B). The qRT-PCR suggested that miR-9-5p inhibition or MEG3 overexpression significantly promoted KLF4 expression, and miR-9-5p overexpression or MEG3 knockdown worked oppositely (Figures 6C–F), indicating that KLF4 expression was negatively regulated by miR-9-5p and positively regulated by MEG3 in chondrocytes.

**FIGURE 6:** KLF4 was the target of miR-9-5p. **(A)** Bioinformatics analysis and luciferase reporter assay confirmed that miR-9-5p could bind to KLF4 3′UTR. **(B)** The expression of KLF4 was decreased in chondrocytes treated with IL-1β. **(C)** After the transfection of miR-9-5p mimic, the expression of KLF4 in chondrocytes was upregulated. **(D)** After the transfection of miR-9-5p inhibitor, the expression of KLF4 in chondrocytes was downregulated. **(E)** After the up-regulation of MEG3 expression, the expression of KLF4 in chondrocytes was upregulated. **(F)** After the down-regulation of MEG3 expression, the expression of KLF4 in chondrocytes was downregulated. Compared with miR-NC, control, pcDNA3.1–NC, or si-NC, **P < 0.01 and ***P < 0.001.

### KLF4 Overexpression Could Counteract the Effects of MEG3 Knockdown on Chondrocytes

We then focused on whether the selective regulation of KLF4 can influence the effects of MEG3 on chondrocytes. The CCK-8 and wound healing assays suggested that, as against the si-MEG3 group, when chondrocytes were co-transfected with pcDNA3.1–KLF4, the viability and migration ability of CHON-001 and ATDC5 cells were significantly enhanced (Figures 7A–C), but the apoptosis and inflammatory reaction were observably repressed (Figures 7D–F). Therefore, it was concluded that the protective effects of MEG3 on chondrocytes were mediated by KLF4.

**FIGURE 7:** KLF4 could counteract the effects of MEG3 knockdown on chondrocytes. **(A–D)** The overexpression of KLF4 could reverse the effects of knocking down MEG3 on the viability, migration, and apoptosis of chondrocytes. (**E**,**F**) The overexpression of KLF4 could reverse the effects of knocking down MEG3 on inflammatory factors, including IL-6, IL-8, and TNF-α. Compared with si-NC, si-MEG3, or si-MEG3 + pcDNA3.1–KLF4, *P < 0.05, **P < 0.01, and ***P < 0.001.

## Discussion

It is reported that more than 200 million people around the world suffered from OA, which can lead to joint pain, stiffness, loss of motor function, and decline in quality of life (Gbd 2016 Disease and Injury Incidence and Prevalence Collaborators, 2017). The molecular mechanism of OA is still indeterminate. Chondrocyte hypertrophy, senescence, and apoptosis are regarded as crucial biological events during the initiation and development of OA (Charlier et al., 2016; Rim et al., 2020). In the present work, it was demonstrated that the MEG3/miR-9-5p/KLF4 axis was involved in regulating the viability, migration, apoptosis, and inflammatory response of chondrocytes.

MEG3 expression is significantly down-regulated in chondrocytes of OA patients, and MEG3 can promote the proliferation of chondrocytes and repress the apoptosis and degradation of extracellular matrix *via* regulating the miR-361-5p/FOXO1 axis (Wang A. et al., 2019). Another study reveals that MEG3 expression is inversely associated with VEGF expression in articular cartilage samples of OA patients, and MEG3 may block OA progression by repressing angiogenesis (Su et al., 2015). These two studies suggest that MEG3 has a protective role for chondrocytes and cartilage, and its defect contributes to the pathogenesis of OA. In the present work, it was authenticated that MEG3 expression was restrained markedly in IL-1β-induced chondrocytes. Furthermore, MEG3 overexpression could strengthen the viability of chondrocytes and suppress apoptosis and inflammation. Conversely, silencing MEG3 led to severer injury of chondrocytes. Our data suggested that the inhibition of MEG3 expression was a pathogenic factor in OA, and the restoration of MEG3 might block or reverse the progression of OA, which is consistent with the two studies mentioned above. Notably, another study also demonstrates that MEG3 expression is significantly declined in the cartilage tissue of OA rat model. However, knocking down MEG3 promotes the proliferation of rat chondrocytes and inhibits apoptosis through the miR-16/SMAD7 axis (Xu and Xu, 2017). This contradictory result may be due to the heterogeneity of different cell models used in different studies, which requires further investigation in the future.

Accumulating studies confirm that miRNAs figure prominently in OA progression. For example, miR-103 expression is significantly increased in the cartilage tissue of OA patients and rat models, and miR-103 can promote OA progression by down-regulating the PI3K/AKT pathway and reducing SPHK1 activity (Li et al., 2019). MiR-146a expression is markedly raised in the OA model induced by IL-1β *in vitro*, and miR-146a can promote the pathogenesis of OA by targeting Smad4 to increase VEGF expression and inhibit the TGF-β signaling pathway (Li et al., 2012). Reportedly, lncRNAs can act as ceRNAs (or molecular sponges) to regulate the activity of miRNAs (Salmena et al., 2011). In the present work, our data implied that MEG3 could probably be a ceRNA for miR-9-5p and repress the expression of miR-9-5p in chondrocytes. According to previous reports, miR-9-5p is a participator in the progression of a variety of tumors. For example, miR-9-5p can target PAK4 to repress the proliferation and inhibit the apoptosis of colon cancer cells (Wang M. et al., 2019); in cervical cancer, miR-9-5p can regulate the angiogenesis and radiosensitivity of cervical cancer cells by targeting SOCS5 (Wei et al., 2019). Interestingly, it is reported that miR-9-5p expression is significantly elevated in the cartilage tissues of OA patients (Kopanska et al., 2017). Herein, consistently, we reported that miR-9-5p was highly expressed in OA models *in vitro*, and additionally, it was found that miR-9-5p could reverse the protective role of MEG3 on chondrocytes, suggesting that miR-9-5p was an injurious factor during OA progression. However, a previous study finds that, in the cartilage of OA mice following tibial plateau fracture, miR-9-5p can suppress chondrocyte apoptosis and promote cartilage remodeling (Chen et al., 2019b), which is different from our study. The reason might be that the previous study constructs a mouse model of traumatic osteoarthritis, while this study used IL-1β to induce OA *in vitro*. The conflicting data suggest that the role of miR-9-5p in OA requires further investigation in future studies.

KLF4 belongs to Sp/KLF family. As a transcription factor, KLF4 is involved in regulating diverse biological processes of cells, such as cell proliferation, differentiation, and apoptosis. Reportedly, KLF4 can regulate bone development and formation by coordinating the differentiation and migration of osteoblasts, osteoclasts, vascular endothelial cells, and chondrocytes (Fujikawa et al., 2014). Besides that, KLF4 expression is significantly down-regulated in ATDC5 cells stimulated by lipopolysaccharide, and this suggests that the down-regulation of KLF4 expression is linked to the inflammatory response of chondrocytes (Fan et al., 2019). Importantly, the expression of KLF4 is repressed in the cartilage of OA patients, indicating that KLF4 is a crucial regulator in OA pathogenesis (Fisch et al., 2018). In the present work, KLF4 was identified as a target gene of miR-9-5p in chondrocytes, and its expression could be positively regulated by MEG3. KLF4 overexpression could partly reverse the viability, migration, apoptosis, and inflammatory response of chondrocytes, which were regulated by MEG3 knockdown. Our study provided a reasonable explanation for the dysregulation of KLF4 in OA. Recently, a study reports that MEG3 can alleviate cerebral I/R injury by binding to KLF4 and inhibit its protein expression (Li et al., 2020), which is inconsistent with our study. The reason may be that MEG3 could exert different functions and specifically regulate the expressions of genes in diverse diseases.

This work has certain limitations. First of all, the conclusion of the present study is based on *in vitro* experiments, and the regulatory function of MEG3 on OA development should be verified with animal models in future studies. Moreover, the downstream mechanism of KLF4 in protecting chondrocytes is still obscure.

To recapitulate briefly, MEG3 can promote chondrocyte viability and migration and restrain apoptosis and inflammation in an OA model *in vitro*. Mechanistically, MEG3 can repress miR-9-5p expression to positively regulate KLF4 expression in chondrocytes. Our study provides a promising target for OA treatment.

## Data Availability Statement

The original contributions presented in the study are included in the article/supplementary material, further inquiries can be directed to the corresponding author/s.

## Author Contributions

YH, XP, and HY conceived and designed the experiments. YH, DC, and ZY performed the experiments. DC, JZ, XX, and XP contributed to the statistical analysis. YH, HY, and XP wrote the manuscript. All authors read and approved the final manuscript.

## Conflict of Interest

The authors declare that the research was conducted in the absence of any commercial or financial relationships that could be construed as a potential conflict of interest.

## References

[B1] CharlierE.RelicB.DeroyerC.MalaiseO.NeuvilleS.ColléeJ. (2016). Insights on Molecular Mechanisms of Chondrocytes Death in Osteoarthritis. *Int. J. Mol. Sci.* 17:2146. 10.3390/ijms17122146 27999417PMC5187946

[B2] ChenH.YangJ.TanZ. (2019a). Upregulation of microRNA-9-5p inhibits apoptosis of chondrocytes through downregulating Tnc in mice with osteoarthritis following tibial plateau fracture. *J. Cell Physiol.* 234 23326–23336. 10.1002/jcp.28900 31169312

[B3] ChenH.YangJ.TanZ. (2019b). Upregulation of microRNA-9-5p inhibits apoptosis of chondrocytes through downregulating Tnc in mice with osteoarthritis following tibial plateau fracture. *J. Cell Physiol.* 234 23326–23336.3116931210.1002/jcp.28900

[B4] DaheshiaM.YaoJ. Q. (2008). The interleukin 1beta pathway in the pathogenesis of osteoarthritis. *J. Rheumatol.* 35 2306–2312. 10.3899/jrheum.080346 18925684

[B5] FanL.LiM.CaoF. Y.ZengZ. W.LiX. B.MaC. (2019). Astragalus polysaccharide ameliorates lipopolysaccharide-induced cell injury in ATDC5 cells via miR-92a/KLF4 mediation. *Biomed. Pharmacother.* 118:109180. 10.1016/j.biopha.2019.109180 31302422

[B6] FischK. M.GaminiR.Alvarez-GarciaO.AkagiR.SaitoM.MuramatsuY. (2018). Identification of transcription factors responsible for dysregulated networks in human osteoarthritis cartilage by global gene expression analysis. *Osteoarthritis Cartilage* 26 1531–1538. 10.1016/j.joca.2018.07.012 30081074PMC6245598

[B7] FujikawaJ.TanakaM.ItohS.FukushiT.KurisuK.TakeuchiY. (2014). Kruppel-like factor 4 expression in osteoblasts represses osteoblast-dependent osteoclast maturation. *Cell Tissue Res.* 358, 177–187. 10.1007/s00441-014-1931-8 24927920

[B8] Gbd 2016 Disease and Injury Incidence and Prevalence Collaborators (2017). Global, regional, and national incidence, prevalence, and years lived with disability for 328 diseases and injuries for 195 countries, 1990-2016: a systematic analysis for the Global Burden of Disease Study 2016. *Lancet* 390 1211–1259.2891911710.1016/S0140-6736(17)32154-2PMC5605509

[B9] GhalebA. M.YangV. W. (2017). Kruppel-like factor 4 (KLF4): What we currently know. *Gene* 611 27–37. 10.1016/j.gene.2017.02.025 28237823PMC5391259

[B10] HeY.LuoY.LiangB.YeL.LuG.HeW. (2017). Potential applications of MEG3 in cancer diagnosis and prognosis. *Oncotarget* 8 73282–73295. 10.18632/oncotarget.19931 29069869PMC5641212

[B11] KapoorM.Martel-PelletierJ.LajeunesseD.PelletierJ. P.FahmiH. (2011). Role of proinflammatory cytokines in the pathophysiology of osteoarthritis. *Nat. Rev. Rheumatol.* 7 33–42. 10.1038/nrrheum.2010.196 21119608

[B12] KopanskaM.SzalaD.CzechJ.GabłoN.GargaszK.TrzeciakM. (2017). MiRNA expression in the cartilage of patients with osteoarthritis. *J. Orthop. Surg. Res.* 12:51. 10.1186/s13018-017-0542-y 28351380PMC5371266

[B13] LeiJ.FuY.ZhuangY.ZhangK.LuD. (2019). LncRNA SNHG1 alleviates IL-1beta-induced osteoarthritis by inhibiting miR-16-5p-mediated p38 MAPK and NF-kappaB signaling pathways. *Biosci. Rep.* 39:BSR20191523. 10.1042/BSR20191523 31383786PMC6732361

[B14] LiF.YaoJ.HaoQ.DuanZ. (2019). miRNA-103 promotes chondrocyte apoptosis by down-regulation of Sphingosine kinase-1 and ameliorates PI3K/AKT pathway in osteoarthritis. *Biosci. Rep.* 39:BSR20191255. 10.1042/BSR20191255 31652455PMC6822578

[B15] LiJ.HuangJ.DaiL.YuD.ChenQ.ZhangX. (2012). miR-146a, an IL-1beta responsive miRNA, induces vascular endothelial growth factor and chondrocyte apoptosis by targeting Smad4. *Arthritis Res. Ther.* 14:R75. 10.1186/ar3798 22507670PMC3446449

[B16] LiT.LuoY.ZhangP.GuoS.SunH.YanD. (2020). LncRNA MEG3 regulates microglial polarization through KLF4 to affect cerebral ischemia-reperfusion injury. *J. Appl. Physiol.* 129 1460–1467. 10.1152/japplphysiol.00433.2020 33180644

[B17] LoeserR. F.GoldringS. R.ScanzelloC. R.GoldringM. B. (2012). Osteoarthritis: a disease of the joint as an organ. *Arthritis. Rheum.* 64 1697–1707. 10.1002/art.34453 22392533PMC3366018

[B18] RimY. A.NamY.JuJ. H. (2020). The Role of Chondrocyte Hypertrophy and Senescence in Osteoarthritis Initiation and Progression. *Int. J. Mol. Sci.* 21:2358. 10.3390/ijms21072358 32235300PMC7177949

[B19] SalmenaL.PolisenoL.TayY.KatsL.PandolfiP. P. (2011). A ceRNA hypothesis: the Rosetta Stone of a hidden RNA language? *Cell* 146 353–358. 10.1016/j.cell.2011.07.014 21802130PMC3235919

[B20] SherwoodJ. (2019). Osteoarthritis year in review 2018: biology. *Osteoarthritis Cartilage* 27 365–370. 10.1016/j.joca.2018.10.005 30808484

[B21] SuW.XieW.ShangQ.SuB. (2015). The Long Noncoding RNA MEG3 Is Downregulated and Inversely Associated with VEGF Levels in Osteoarthritis. *Biomed. Res. Int.* 2015:356893. 10.1155/2015/356893 26090403PMC4454735

[B22] SwinglerT. E.WheelerG.CarmontV.ElliottH. R.BarterM. J.Abu-ElmagdM. (2012). The expression and function of microRNAs in chondrogenesis and osteoarthritis. *Arthritis. Rheum.* 64 1909–1919. 10.1002/art.34314 22143896

[B23] TanakaM.ItohS.FukushiT.KurisuK.TakeuchiY.MorisakiI. (2014). Kruppel-like factor 4 expression in osteoblasts represses osteoblast-dependent osteoclast maturation. *Cell Tissue Res.* 358 177–187. 10.1007/s00441-014-1931-8 24927920

[B24] TayY.RinnJ.PandolfiP. P. (2014). The multilayered complexity of ceRNA crosstalk and competition. *Nature* 505 344–352. 10.1038/nature12986 24429633PMC4113481

[B25] WangA.HuN.ZhangY.ChenY.SuC.LvY. (2019). MEG3 promotes proliferation and inhibits apoptosis in osteoarthritis chondrocytes by miR-361-5p/FOXO1 axis. *BMC Med. Genomics* 12:201. 10.1186/s12920-019-0649-6 31888661PMC6937924

[B26] WangM.GaoQ.ChenY.LiZ.YueL.CaoY. (2019). PAK4, a target of miR-9-5p, promotes cell proliferation and inhibits apoptosis in colorectal cancer. *Cell Mol. Biol. Lett.* 24:58. 10.1186/s11658-019-0182-9 31728150PMC6842216

[B27] WeiY. Q.JiaoX. L.ZhangS. Y.XuY.LiS.KongB. H. (2019). MiR-9-5p could promote angiogenesis and radiosensitivity in cervical cancer by targeting SOCS5. *Eur. Rev. Med. Pharmacol. Sci.* 23 7314–7326.3153911810.26355/eurrev_201909_18837

[B28] XuJ.XuY. (2017). The lncRNA MEG3 downregulation leads to osteoarthritis progression via miR-16/SMAD7 axis. *Cell Biosci.* 7:69. 10.1186/s13578-017-0195-x 29255591PMC5727780

[B29] ZhiL.ZhaoJ.ZhaoH.QingZ.LiuH.MaJ. (2020). Downregulation of LncRNA OIP5-AS1 Induced by IL-1beta Aggravates Osteoarthritis via Regulating miR-29b-3p/PGRN. *Cartilage* 2020:940077951. 10.1177/1947603519900801 32037864PMC8804817

